# Mismatch repair status between primary colorectal tumor and metastatic tumor, a retrospective consistent study

**DOI:** 10.1042/BSR20190730

**Published:** 2019-12-13

**Authors:** Zheng Wang, Xiaoli Tang, Xiaoqing Wu, Meiyuan Yang, Daorong Wang

**Affiliations:** 1 Department of General Surgery, Northern Jiangsu Province Hospital, Clinical Medical College, Yangzhou University, Institute of General Surgery—Yangzhou, Yangzhou, P.R. China; 2 Department of General Surgery, The Second Xiangya Hospital of Central South University, Changsha, P.R. China

**Keywords:** Colorectal cancer, Immunohistochemistry, immunotherapy, Mismatch repair

## Abstract

**Objectives** Mismatch repair (MMR) and Microsatellite instability (MSI) are critical when considering immunotherapy and chemotherapeutic drugs an option for patients with colorectal cancer (CRC). We investigated the consistence of MMR status as well as MSI between primary CRC and metastatic tumor to see if the expression of four MMR proteins and the status of MSI are congruent in primary tumor and metastatic tumor. With the results of the study and future more relevant studies, the sites of MMR testing may be more precise for individualized treatment.

**Study design** Patients with clear diagnosis of sporadic CRC and distal organ metastasis were identified from a prospectively established database. The status of MMR and MSI was evaluated by immunohistochemistry (IHC) and Polymerase Chain Reaction (PCR) respectively of synchronously obtained tissue samples.

**Results** Forty patients with complete clinical date were enrolled. For primary tumor, 36/40 samples were tested as MMR-proficient (pMMR) and 4 were MMR-deficient (dMMR). For metastatic samples, 30 samples were tested as pMMR while 10 samples were dMMR. Six out of forty patients were tested as inconsistent status of MMR and MSI. After statistical analysis, the expression status of MMR was not statistically significant between primary and metastatic tumors (*P*=0.1405, larger than 0.05).

**Conclusion** Based on our samples, the status of MMR between primary CRC and metastatic tumor was consistent, thus test of MMR status can be performed at both sites. However, due to the limited samples enrolled in our study, the results should be interpreted carefully.

## Introduction

Colorectal cancer (CRC) is one of the leading neoplasm around the world with more than 10000 new cases diagnosed per year in the United States [1]. Approximately 21% of CRC was metastatic and estimated 5-year survival for these patients was 13.9% [1,2]. The liver is the most common site for metastatic CRC and previously reported 3-year disease-free survival is approximately 14% after a hepatic resection [3]. Most of cases diagnosed with liver metastasis are unresectable and the first-line therapy for them was chemotherapy [4,5]. Mismatch Repair (MMR) Gene is defined as functional recognizing and repairing DNA damage during duplication [6]. Mutation of MMR gene usually results in loss of MMR protein and thus the tumor DNA becomes microsatellite instability-high (MSI/MSI-H) which leads to numerous mutations within the tumor cell [7]. CRC with MMR mutation was considered as a specific subtype of CRC which has distinct clinicopathologic features like proximal location, right-sided tumor, low metastasis and longer survival in early stage [8–10].

Recent studies suggested that the status of patients’ status of MMR or MSI could be a predictive biomarker to assess whether they can benefit from PD-1 immune checkpoint inhibitory therapy [11,12]. Evidence suggested that patients with MMR-deficient (dMMR) or MSI-H had higher objective response rate and longer progression-free survival compared with MMR-proficient (pMMR) or Microsatellite stable (MSS) patients after receiving immunotherapy [13,14]. Therefore, the status of MMR could be crucial when considering immune therapy as a treatment option [15,16]. In addition, previous studies have shown that the mutation status of K-Ras was congruent between primary tumor and metastasis lesion so the NCCN guideline 2017 suggested that testing of K-Ras can be performed at both primary and metastatic lesion [17–19]. However, few studies have focused on consistency of MMR status between primary CRC and matching liver metastasis lesions especially without neoadjuvant chemotherapy before the testing [20]. Therefore, we did a consistency study between primary tumor and matching liver metastasis lesion through immunohistochemistry (IHC) and Polymerase Chain Reaction (PCR) to determine the congruence of MMR and MSI status between primary tumor and metastatic lesion.

## Materials and methods

Consecutive patients who underwent metastatic resection or biopsy for CRC metastases at Northern Jiangsu Province Hospital from 2015 to 2017 were identified. The inclusion criteria were as following: stage IV CRC with pathological confirmation, available samples of both primary and metastatic lesions, complete records of clinical data and follow-up information. Any previous malignancy history other than CRC patients underwent liver transplantation before and patients went through adjuvant chemotherapy were excluded from the study. Informed written consents were obtained from all enrolled patients and the nature of the study was explained by physicians to all patients enrolled.

### IHC

Formalin-fixed, paraffin-embedded blocks of primary cancer tissue and matching metastatic lesions were prepared for IHC. The samples were deparaffinized after washing in xylene, graded alcohol and distilled water. Then 3% H_2_O_2_ was used to block the activity of endogenous peroxidase and antigen was retrieved by boiling the samples twice for 3 min each time. Non-specific protein binding was blocked by embedded with 10% goat serum at 37°C for half an hour. The following primary antibodies were used for staining, MLH1 (dilution; 1:200, Abcam, U.K.), MSH2 (dilution; 1:200, Cell Signaling Technology, U.S.A.), MSH6 (dilution, 1:500, Cell Signaling Technology, U.S.A.), PMS2 (dilution; 1:200, Abcam, U.K.). The samples were visualized using a DAB kit and counterstained by Hematoxylin. Any nuclear staining of tumor cell was defined as positive thus the slide was tested as protein positive. Complete loss of detectable staining of the nucleus was defined as protein deficient and any type of the four protein loss was referred as dMMR [21]. The staining was assessed by two experienced pathologists who were blinded to the clinical data of the patients. To objectively assess the staining of the slides, we also used ImageJ (Version 1.51w, NIH) to calculate the area of staining by regulating the gray-scale value of the slides to separate positive staining from the background. Finally, if the results from the pathologists contradict the results from ImageJ, we used Image-Pro Plus, a commercial software specializing in processing images, to assess the slides.

### MSI-PCR

MSI-PCR was performed by using the Colorectal Cancer Microsatellite Instability Testing Kit (MicroRead, Beijing, China) under the manufacturer’s instructions. Briefly, DNA was extracted from paraffin embedded samples and amplified following the instructions. Based on comparison of the mentioned mononucleotides’ markers, MSI was defined as one unstable marker (MSI-low) and two or more as MSI-high while MSS was identified as no unstable marker [22]. The Applied Biosystems 9700 and the Applied Biosystems 3730xl were used for PCR and genetic analysis.

### Statistics analyses

Clinical characteristics including age, gender, pathology diagnosis, TNM staging and lymph nodes involvement were retrospectively collected from the database. Correlation between primary MMR status and metastatic lesion were analyzed using Fisher exact and χ^2^ tests. All statistical analyses were performed through SPSS Version 23 (IBM Corp., Armonk, NY, U.S.A.) with a significance level of *P*<0.05.

## Results

### Clinical data

There were 40 patients enrolled in the present study with a mean age of 58.5 years. The clinical characteristics and status of consistency between primary tumor and metastatic tumor are summarized in Table 1. No cancerous family history was found within these patients. Lymph node metastasis was found to be associated with inconsistent status of MMR.

**Table 1:** Clinical characteristics of enrolled patients

Variable	Number of patients	Consistent expression of MMR	Inconsistent expression of MMR	*P*-value
Age				
<60	22	16	6	0.4761
≥60	18	15	3	
Gender				
Male	24	18	6	0.6428
Female	16	13	3	
Tumor location				
Left	31	25	6	0.3941
Right	9	6	3	
Differentiation				
Well/Moderate	34	25	9	
Poor	6	6	0	0.3065
T stage				
Non-T4	13	10	3	>0.9999
T4	27	21	6	
Lymph node metastasis				
Yes	15	15	0	0.0151*
No	25	16	9	

*P ≤ 0.05 The difference is statistically significant.

### MMR status

All resections were estimable after staining. The result evaluated by pathologists were not contradictive with the results from ImageJ. For primary tumor, four slides were defined as dMMR and the rest of the samples as pMMR. For metastatic lesion, 10 of 40 samples were dMMR while 30 of them were pMMR. Thirty cases were tested both pMMR in primary and metastatic tumors. Four cases were both dMMR in primary and metastatic tumors. Six cases were pMMR in primary tumor while dMMR in metastatic tumor. After Fisher’s exact test of the data (shown in Figure 1), the occurrence of dMMR was found not significantly different between primary and metastatic tumors, as it is shown in Figure 1. Typical examples of expression and loss of expression of MLH1 were shown in Figure 2A–D.

**Figure 1:** Analysis of consistence of MMR status of primary and metastatic tumors

**Figure 2:** MLH1 protein expression in primery and metastatic tumor (**A**) MLH1 protein expression in primary tumor. (**B**) Loss of MLH1 protein expression in primary tumor. (**C**) MLH1 protein expression in metastatic tumor. (**D**) Loss of MLH1 protein expression in metastatic tumor.

### MSI status

After testing for MSI status by PCR, the four dMMR samples in primary tumor tested by IHC were identified as MSI-high by PCR as well as the ten dMMR samples from metastatic tumor. As it was shown in Figure 3A,B, we tested six mononucleotide repeats (NR-27, NR-28, Bat-25, Bat-26, NR-24, Mono-27) and pentanucleotide markers (Penta C, Penta D) and Amel in each pair of primary and corresponding metastatic tumors. The results of MSI testing were concordant with IHC.

**Figure 3:** Testing for MSI status by in pentaplex PCR in primary and metastatic tumor (**A**) Microsatellite Stable. (**B**) Microsatellite Instable.

## Discussion

The status of MMR expression has a significant role in deciding the use of immunotherapy, especially when first-line chemotherapy has failed in advanced CRC. Clinical trial conducted by Le et al. [13] published in *New England Journal of Medicine* in 2015 demonstrated that patients with dMMR benefited more from PD-1 therapy. In the NCCN Clinical Practice Guidelines for CRC, PD-1 therapy was recommended for patients with dMMR status [23]. However, there is no clear conclusion about whether is it necessary to test MMR at both primary and metastatic lesion or not.

In the present study, we studied the expression status of MMR and MSI in primary CRC and corresponding metastatic liver tumor. Based on our results, expression of MMR was lost in 10% primary tumor and 25% in liver metastasis. Existing studies have tried to explore the correlation between primary and metastatic tumors regarding MMR expression. Jung et al. [24] did their consistency study between primary and metastatic lesions with a 77% consistence. However, the metastatic samples they used were obtained after adjuvant chemotherapy. It is still under great debate about whether using chemotherapy will change the status of MMR expression which means the results from Jung et al. may be influenced by this potential confounding factor [25,26]. Our results also indicated that inconsistent expression of MMR was related to lymph node metastasis. Previous studies have reported that dMMR was not related to positive lymph node metastasis [27]. Unfortunately, our limited samples failed to further investigate the correlation between subtype of inconsistent expression of MMR in primary and metastatic tumors and lymph node invasion.

The Current NCCN Clinical Practice Guideline recommended testing of MMR in CRC patients diagnosed at age ≤70 years. However, there was no recommendation about where the testing should be applied. When it comes to test RAS mutation for therapy advice, previous evidence has demonstrated the consistency of RAS mutation between primary tumor and metastatic tumor [28,29], thus the guideline recommended testing to be taken at primary or metastatic sites. However, no recommendation was made concerning the location of testing for MMR in CRC. Based on our result, due to the consistency of MMR status between primary and liver metastatic tumors, testing can be made at primary or liver metastatic lesions.

Our study has some certain limitations. First, the size of our patients sample is still too small to confirm a more widespread conclusion. Second, due to the difficulty of multisampling, our only tested one site instead of five sites for each patient. Studies have reported intratumoral heterogeneity thus the results from our study may be occasional [30,31].

The strength of our study is that we used the samples from simultaneous resection without any previous chemotherapy, which means the status of MMR or MSI was not affected by the chemotherapeutics. Our study formed a preliminary conclusion that MMR expression was consistent between primary CRC and corresponding liver metastasis.

## Conclusion

The MMR or MSI status between primary CRC and liver metastasis is consistent according to our center’s data. Therefore, when considering immunotherapy or evaluating individual prognosis of an advanced CRC patient, testing of MMR can be taken place at primary tumor or liver metastatic lesion.

## Informed Consent

Informed consent was obtained from all individuals participants enrolled in the study.

## Abbreviations

CRC: colorectal cancer
DAB: Diamobenzidine
dMMR: MMR-deficient
IHC: immunohistochemistry
MLH1: MutL protein homolog 1
MMR: mismatch repair
MSH2: MutS protein homolog 2
MSI: microsatellite instability
MSI-H: MSI-high
MSS: microsatellite stable
PCR: polymerase chain reaction
PD-1: Programmed cell death protein 1
pMMR: MMR-proficient
PMS2: PMS1 protein homolog 2
RAS: Rat sarcoma
TNM: Tumor Node metastasis
